# Primary Small Cell Undifferentiated (Neuroendocrine) Carcinoma of the Maxillary Sinus

**DOI:** 10.1155/2014/463109

**Published:** 2014-02-03

**Authors:** Santosh Kumar Yadav, Premalatha Shetty

**Affiliations:** ^1^Department of Oral and Maxillofacial Surgery, Chitwan Medical College (P) Ltd, P.O. Box 42, Bharatpur-10, Chitwan, Nepal; ^2^Department of Oral and Maxillofacial Surgery, Manipal College of Dental Sciences, Manipal University, Lighthouse Hill Road, Mangalore 575001, India

## Abstract

Primary small cell neuroendocrine carcinoma (SNEC) of the paranasal sinuses is an extremely rare and distinctive tumor with aggressive clinical behavior. Moreover, SNECs originating in the head and neck region have been reported to be highly aggressive and to have a poor prognosis. This report describes a patient with a maxillary sinus SNEC who was successfully treated with neoadjuvant chemotherapy and concurrent chemoradiotherapy.

## 1. Introduction

Carcinoma developing in the paranasal sinuses accounts for approximately 0.3% of all cancers [1]. Squamous cell carcinoma is by far the most common malignancy, followed by adenocarcinoma. Extrapulmonary small cell neuroendocrine carcinoma (EPSNEC) of sinonasal tract is rare. The first case of SNEC of the paranasal sinuses was reported by Raychowdhuri [2] in 1965. SNECs originating in the head and neck region have been reported to be highly aggressive and to have a poor prognosis. This report describes a patient with a maxillary sinus SNEC who was successfully treated with neoadjuvant chemotherapy and concurrent chemoradiotherapy. The clinical and pathologic features of the tumor and the optimal treatment of this patient are discussed.

## 2. Case Report

A 70-year-old female presented to the oral and maxillofacial department with gradual onset of right cheek swelling around the right gingival and a painful mass for about 1 month. Physical examination showed hard cheek swelling (Figure 1) and epiphora of the right eye, but the patient's eye movement was normal and she did not have any double vision. The skin around the right eyelids was regular and not reddish, whereas the right posterior alveolar gingival was ulceration (2 × 2) cm, irregular, and reddish in areas (Figure 2). No history of nasal bleed, nasal congestion, and pus from ears. Clinically the patient had an enlarged right submandibular lymph node measuring approximately 3 cm in diameter. The patient was admitted, and imaging studies were performed.

Computed tomography (CT) scan of head showed a large mass measuring approximately 6 cm in diameter in the right maxillary sinus invading the right orbit, ethmoid sinus, and the skin of the cheek (Figures 3(a) and 3(b)). Histologic examination of biopsy sample stained sections showed mucosal tissue bits with features suggestive of poorly differentiated squamous cell carcinoma/neuro-endocrine carcinoma and immunohistochemistry was advised for further evaluation. Immunohistochemical staining was performed on the formalin-fixed, paraffin-embedded tissue sections. The tumor cells were positive for synaptophysin and cytokeratin and negative for neuron specific enolase. These histologic (Figure 4) and immunophenotypic features were characteristic of SNEC, and clinical findings supported the diagnosis of small cell undifferentiated neuroendocrine carcinoma of right maxillary sinus. An extensive search for a primary lesion elsewhere was performed; however, findings from whole body CT imaging, urinary amine secretions, and sputum cytology were unremarkable.

This case was discussed with consulting medical and radiation oncologists and planned for combination of chemotherapy followed by radiotherapy. The patient was treated with 3 cycles of induction chemotherapy, consisting of cisplastin (40 mg/m^2^) and etoposide (100 mg/m^2^) on days 1 to 3 every 4 weeks. After induction chemotherapy, it was extremely effective, with remarkable reduction in facial swelling and complete loss of intraoral swelling (Figures 5 and 6). The patient was subsequently started on concurrent chemoradiation, consisting of 1 course of cisplastin and etoposide similar to the induction chemotherapy, and a total dose of 60 Gy of intensity modulated radiation therapy in 30 fractions, 5 days a week for a total of 6 weeks. The patient's posttherapeutic course was uneventful. Follow-up 2-year postradiotherapy showed no evidence of local recurrence or metastasis (Figures 7, 8, and 9).

## 3. Discussion

SNEC occurs mainly in lungs and accounts for approximately 20% of primary lung carcinomas [3]. EPSNEC represents 4% of all cases of SNEC [4], and a limited number of SNEC cases of the nasal and paranasal cavities have been previously reported. Among these tumors, primary SNEC arising in the maxillary sinus is extremely rare. The classification of neuroendocrine tumor is particularly difficult, as indicated by several investigators [5]. Carcinoid tumor is considered a well-differentiated neuroendocrine carcinoma, although atypical carcinoid tumor is regarded as moderately differentiated neuroendocrine carcinoma. SNEC is classified as poorly differentiated neuroendocrine carcinoma. Similar to SNEC of the lung, SNEC of the nasal and paranasal cavities has demonstrated aggressive clinical behavior and a poor prognosis, with fast tumor expansion, early local recurrence, and widespread dissemination.

As originally described by Koss et al. [6] and Georgiou et al. [7], SNEC of all anatomic sites shares similar histopathologic features. The tumor forms sheets or nests and is composed of medium-sized tumors cells with a high nuclear/cytoplasmic ratio and hyperchromatic nuclei with indistinct or occasional small basophilic nucleoli.

According to criteria of the World Health Organization [8], small cell carcinomas are defined as malignant epithelial tumors consisting of small cells with scant cytoplasm, ill-defined cell borders, finely granular nuclear chromatin, and absent or inconspicuous nucleoli. Specific cells are round, oval, and spindle shaped, and nuclear molding is prominent. Necrosis is usually extensive, and the mitotic count is high. More than 90% of small cell carcinomas have neuroendocrine features [8].

The immunohistochemical tumor profile has been previously investigated [1, 9] and has demonstrated that the tumor is usually strongly positive for synaptophysin and CD56 and weakly positive for chromogranins and CAM5.2/AE1. The present patient showed positive staining for synaptophysin, indicating that the tumor was of neuroendocrine origin. Tumor cells also were positive for cytokeratin, indicating that the tumor originated from the epithelium.

Because of the rarity of SNEC of the nasal and paranasal cavity, no agreement for adequate management has been reached among oncologists; therefore, much information has been extrapolated from data on SNECs at other sites, especially pulmonary SNECs (PSNECs). Because SNEC is an aggressive malignancy with high rates of local recurrence and metastatic spread, multimodal therapy is increasingly used, including chemotherapy, radiotherapy, and possibly surgery, depending on the extent of disease or the primary site. Since the late 1990s, the combination of chemotherapy and radiotherapy, with or without surgery, has been recommended [10, 11]. The largest study to date tested platinum-based chemotherapy followed by radiotherapy [11]. The chemotherapeutic regimens used for patients with EPSNEC are similar to those used for patients with PSNEC, with the combination of etoposide and cisplastin being the first-line treatment and yielding a response rate of 69% [12]. Radiotherapy also has been shown to be curative at many sites, although the histologic similarity of SNEC of the nasal and paranasal sinuses to PSNEC has suggested that chemotherapy should be the first option. The best method for integrating chemotherapy and head and neck radiotherapy remains unknown. The chemoradiotherapy regimen for the present patient consisted of 4 cycles of cisplastin plus etoposide chemotherapy concurrent with 60 Gy of locoregional radiation administered once or twice daily. Although introduced for the treatment of lung cancer in the late 1970s [13], the combination of cisplastin and etoposide emerged as primary therapy only in the early 1980s [14]. A clear advantage of cisplastin plus etoposide is that this combination can be given concurrently with relatively full doses of thoracic radiotherapy, with lower morbidity rates than observed with doxorubicin-based [15] or cyclophosphamide-based [16] regimens.

The higher rate of intracranial metastases in patients with SNEC of the nasal and paranasal sinuses than in those with PSNEC suggests that patients with the former should be treated with systemic chemotherapy and radiotherapy and prophylactic cranial irradiation [17]. Recurrence and metastasis of SNEC of the nasal and paranasal sinuses during 3 years of follow-up have been reported in up to 70% of patients [18], with an overall local recurrence rate of 33% and a metastasis rate of 31% [19]. The 1- and 5-year survival rates have been reported to be approximately 57% and 10%, respectively, and comparable to rates in patients with EPSNEC, with a 5-year survival rate of 13% and a median survival of 13 months [20]. With the present management strategy, local failure remains an important problem. However, until what governed failure has been appreciated, the surgeon and the oncologist should try to optimize the treatment for each patient with improved local therapy. This may contribute to local control and survival so that cure will be achieved with minimal morbidity. More extensive studies are needed to assess the optimal management and develop standardized treatment protocols.

## Figures and Tables

**Figure 1:** Preoperative right cheek swelling.

**Figure 2:** Preoperative intraoral swelling and ulceration.

**Figure 3:** Imaging analysis. (a) Initial coronal section computed tomography of head showing mass in the right maxillary sinus invading the right orbit, ethmoid sinus. (b) Initial enhanced axial computed tomography of head showing complete destruction of the anterior wall of the maxillary sinus.

**Figure 4:** Histologic findings of biopsy tissue. The tumor was composed of small round to oval hyperchromatic nuclei with dense chromatin and scanty cytoplasm.

**Figure 5:** Chemotherapy after 4th cycle, remarkable reduction in facial swelling.

**Figure 6:** Chemotherapy after 4th cycle, complete loss of intraoral swelling.

**Figure 7:** Follow-up 2-year postradiotherapy.

**Figure 8:** Follow-up 2-year postradiotherapy.

**Figure 9:** Follow-up 2-year CT image.
